The article "Dose Prediction Models Based on Geometric and Plan Optimization Parameter for Adjuvant Radiotherapy Planning Design in Cervical Cancer Radiotherapy" was retracted in 2023. Reasons: unreliable results or conclusions; concerns about the data; concerns about the peer review; concerns about the citations.

# Dose Prediction Models Based on Geometric and Plan Optimization Parameter for Adjuvant Radiotherapy Planning Design in Cervical Cancer Radiotherapy

**DOI:** 10.1155/2021/7026098

**Published:** 2021-11-12

**Authors:** Hui Tang, Yazheng Chen, Jialiang Jiang, Kemin Li, Jing Zeng, Zhenyao Hu, Rutie Yin

**Affiliations:** ^1^Department of Obstetrics and Gynecology, West China Second University Hospital, Sichuan University, Chengdu, China; ^2^Key Laboratory of Birth Defects and Related Diseases of Women and Children (Sichuan University), Ministry of Education, Chengdu, China

## Abstract

The prediction of an additional space for the dose sparing of organs at risk (OAR) in radiotherapy is still difficult. In this pursuit, the present study was envisaged to find out the factors affecting the bladder and rectum dosimetry of cervical cancer. Additionally, the relationship between the dose-volume histogram (DVH) parameters and the geometry and plan dose-volume optimization parameters of the bladder/rectum was established to develop the dose prediction models and guide the planning design for lower OARs dose coverage directly. Thirty volume modulated radiation therapy (VMAT) plans from cervical cancer patients were randomly chosen to build the dose prediction models. The target dose coverage was evaluated. Dose prediction models were established by univariate and multiple linear regression among the dosimetric parameters of the bladder/rectum, the geometry parameters (planning target volume (PTV), volume of bladder/rectum, overlap volume of bladder/rectum (OV), and overlapped volume as a percentage of bladder/rectum volume (OP)), and corresponding plan dose-volume optimization parameters of the nonoverlapping structures (the structure of bladder/rectum outside the PTV (NOS)). Finally, the accuracy of the prediction models was evaluated by tracking *d* = (predicted dose-actual dose)/actual in additional ten VMAT plans. *V*_30_, *V*_35_, and *V*_40_ of the bladder and rectum were found to be multiple linearly correlated with the relevant OP and corresponding dose-volume optimization parameters of NOS (regression *R*^2^ > 0.99, *P* < 0.001). The variations of these models were less than 0.5% for bladder and rectum. Percentage of bladder and rectum within the PTV and the dose-volume optimization parameters of NOS could be used to predict the dose quantitatively. The parameters of NOS as a limited condition could be used in the plan optimization instead of limiting the dose and volume of the entire OAR traditionally, which made the plan optimization more unified and convenient and strengthened the plan quality and consistency.

## 1. Introduction

Cervical cancer (CC) is one of the most common malignant carcinomas among women worldwide and remains the fourth most common cancer worldwide. It is even more common in the low- and middle-income countries, where it appears to be in the second position after breast cancer [1, 2].

The article "Dose Prediction Models Based on Geometric and Plan Optimization Parameter for Adjuvant Radiotherapy Planning Design in Cervical Cancer Radiotherapy" was retracted in 2023. Reasons: unreliable results or conclusions; concerns about the data; concerns about the peer review; concerns about the citations.

Surgery, radiotherapy, and chemotherapy are the main treatments for cervical cancer [3, 4]. Radiotherapy plays a crucial role in the treatment of cervical cancer. Currently, approximately 80% of cervical cancer patients require radiotherapy [5, 6]. To minimize the potential side effects during and after treatment, such as radiation cystitis and radiation enteritis, the dosimetric sparing of the bladder and rectum becomes essential. Radiotherapy toxicity of the bladder and rectum is related to the radiation dose received and the irradiation volume. Studies have also demonstrated that the middose region (>30 Gy) can lead to rectal bleeding [7–11]. Marks et al. found that the majority of the bladder could be irradiated with a dose of approximately 30–50 Gy [12]. When the bladder dose approached 50–60 Gy, the risk of bladder dysfunction begins to increase and severe urinary toxicity might be encountered. Based on the previous studies [13–17], it was observed that, in the bladder and rectum of cervical cancer, the exposure radiation volumes were generally administered in the middose region in the external beam radiotherapy (EBRT). The lower the dose of EBRT to the organs at risk (OAR), the more the dose space of the OARs in brachytherapy in cervical cancer.

Balancing the target's dose and protection of the OAR is still a difficult problem to be solved. There are few methods to determine, whether there is room for more dose reduction of the OARs without losing the dose of the target. Some studies [18–21] found out the relationship between the dose and the geometric parameters of OAR for predicting the dose before planning, but they could not be directly used to guide the plan design. It is known that the experience of the treatment planner largely affects the plan quality, as evident from the large differences in plan quality among planners and different institutes [22]. At present, the design of the radiotherapy plan is still a trial-and-error process of repeated optimization and modification, and the quality of the plan largely depends on the experience of the physiologist and radiotherapy physician that requires a huge amount of time and effort. Although the new era is of automated planning, there remains a need to develop a simple clinician-oriented metric to aid the recognition of plans that struggle to meet the OAR dose constraints directly and improve the quality and efficiency of radiotherapy plan design.

The article "Dose Prediction Models Based on Geometric and Plan Optimization Parameter for Adjuvant Radiotherapy Planning Design in Cervical Cancer Radiotherapy" was retracted in 2023. Reasons: unreliable results or conclusions; concerns about the data; concerns about the peer review; concerns about the citations.

The final dose after plan optimization is easily influenced by many factors in the actual plan optimization process; especially, the different plan designers use different irregular plan optimization parameters, which makes the planning optimization process difficult to control and adjust. Traditional plan optimization parameters often limit the dose volume of the entire OAR, mainly relying on personal experience. Planners, especially young planners with low planning design levels, need to constantly try to find the adaptive plan optimization parameters for their own use. It takes time and effort and results in large differences in the quality of plans between different organizations and planners. In addition, in the case of overlap between OAR and target, it is difficult to balance the dose of target and OAR by dose-volume restriction for the entire OAR. Once the planning parameters are improperly designed, it is easy to make the dose loss in the target area or the protection of OAR is insufficient. And target volume, OAR volume, and their overlapping volume vary from person to person; traditional similar dose-volume optimization parameters of entire OAR are not appropriate. It cannot adjust plans quantitatively and regularly in the process of plan optimization, which still depends on the personal experience and reduces the flexibility and convenience of plan optimization.

In order to find out the influencing factors of OAR dose for meeting the target dose while maximizing the protection of the OAR and make planning optimization more flexible and convenient for improving plan design efficiency and plan quality and homogeneity, the present study employed the bladder/rectum region of the nonoverlapping target area as a structure and the dose limit of this structure was applied in the optimization of the plan instead of traditional plan optimization parameters of entire OARs. The dose-volume parameters of nonoverlapping structure in the study can be as plan optimization parameters. Unlike traditional plan optimization parameters, the dose limits mainly apply to the nonoverlapping structure instead of the entire OAR. In principle, the dose limits do not act on the overlapping area, so as to minimize the dose loss of target for the protection of OAR (unless the doctor requires that some target dose be discarded for the protection of OAR). These parameters can also be used as plan optimization parameters to directly participate in and guide the plan optimization, but no relevant literature has studied the role of this factor and its clinical practicality in the past.

In the high-quality radiotherapy plan, the visible dose falls uniformly outside the target, the interval gradient between different dose lines is similar, and the dose distribution is regular, which can be used to judge whether there is still space for the protection of OAR. Based on this, the nonoverlapping structure is located outside the target, we assume there is regular dose distribution in the nonoverlapping structure, combining with overlapping volume of OAR to study the dose effects on the entire OAR. Because each patient's overlapping volume is fixed, the impact of dose distribution of nonoverlapping structure on the dose of entire OAR cannot be ignored, and the dose distribution in this region can be adjusted, which makes planning optimization more convenient and flexible and its clinical practicability and operability stronger. The aim of this study was to develop a model-based method for prediction of the bladder and rectum dose based on the geometric and radiotherapy planning parameters in cervical cancer radiotherapy. The study was structured in two parts: the first part focused on determining the factors affecting the bladder/rectum dose to develop the models, by retrospectively studying the volumetric-modulated arc therapy (VMAT) plans of 30 patients. The second part verified the feasibility and accuracy of the forecasting models in 10 patients.

The article "Dose Prediction Models Based on Geometric and Plan Optimization Parameter for Adjuvant Radiotherapy Planning Design in Cervical Cancer Radiotherapy" was retracted in 2023. Reasons: unreliable results or conclusions; concerns about the data; concerns about the peer review; concerns about the citations.

## 2. Materials and Methods

### 2.1. Patients and VMAT Plans

A total of forty patients, who underwent VMAT postoperative irradiation for uterine cervical cancer at our hospital, were included in this study. All patients received their first radiotherapy and there were no contraindications to the administered radiotherapy. Thirty plans were randomly selected for modeling and ten patients were selected to verify the accuracy of the model. All the radiotherapy plans were made by the most experienced physiologist in our institution, with a rich experience in radiotherapy planning. The prescribed dose was 50.4 Gy/28 Fr.

VMAT plans were designed by the Varian Treatment Planning System (Eclipse TPS, Version 15.5, Germany). Two gantry rotation angles (2 arcs), 181°∼179° in the clockwise direction and 179°∼181° in the counterclockwise direction, were used for the VMAT. The gantry rotation speed and dose per gantry angle degree were optimized for a variable dose rate plan with a maximum dose rate of 600 MU/min. The dose calculation model was the anisotropic analytical algorithm using a grid size of 0.25 cm × 0.25 cm × 0.25 cm with heterogeneity correction applied. Patients were treated with 6 MV photon with the Trilogy linear accelerator (Varian Medical Systems, Germany).

### 2.2. Planning Evaluation

The dose-volume histograms and dose distributions of each plan were reviewed to ensure the target coverage and OAR sparing. The standard for the acceptance of the plan was that at least 95% volume of the PTV received the prescription dose (*V*_dose_ >95%); meanwhile, the maximal dose (*D*_max_) of the PTV should be <110% of the prescription dose and limited within PTV. OAR dose limits were as follows: bladder V_40_ < 40%, rectum V_40_ < 40%, intestine V_30_ < 40%, and bone V_40_ < 5%. Dose constraints were determined by our institute's treatment directives, which follow the institution request, literature experience, RTOG0418 guidelines [15], and QUANTEC related reports [16, 17]. These parameters were associated with the incidence of adverse reactions in the OAR and were often used as planning evaluation parameters.

The article "Dose Prediction Models Based on Geometric and Plan Optimization Parameter for Adjuvant Radiotherapy Planning Design in Cervical Cancer Radiotherapy" was retracted in 2023. Reasons: unreliable results or conclusions; concerns about the data; concerns about the peer review; concerns about the citations.

### 2.3. Data Collection

The data used to develop the dose prediction models were collected by one physicist. Forty plans data were retrieved to collect the doses to 98%, 95%, 50%, and 2% of the PTV (*D*_98_, *D*_95_, *D*_50_, and *D*_2_) according to the International Commission on Radiation Units and Measurements Report No. 83 [23] for target dose assessment. In addition, the conformal index (CI) and homogeneity index (HI) for PTV were calculated. The formula of CI defined as CI=*V*_*T*,ref_/*V*_*T*_*∗V*_*T*,ref_/*V*_ref_, *V*_*T*,ref_ is the volume of target, where the received dose is equal to or greater than the reference dose, cm^3^; *V*_T_ is the volume of target, cm^3^; *V*_ref_ is the volume at which the received dose is equal to or greater than the reference dose, cm^3^. CI ranges from 0 to 1. CI = 1, indicating that the reference dose accurately covers the target volume, the healthy tissue is not irradiated above the prescribed dose, and the conformation is the best. CI = 0, indicating that there is no conformal, and the conformal is the worst [24–26]. HI = (*D*_2_−*D*_98_)/*D*_50_, wherein according to ICRU 83 report, *D*_2_ and *D*_98_ represent the near-maximum dose and the near-minimum dose, respectively [23]. The higher the CI value, the better the conformability of the dose to the target area. The smaller the HI value (closer to 0), the better the uniformity of the target dose. For the bladder and rectum, dosimetric outcome measures included the 2 cm^3^ maximum dose (*D*_2cc_), percentage of volume receiving a dose of ≥30 Gy (*V*_30_), 35 Gy (*V*_35_), and 40 Gy (*V*_40_) and these dosimetric parameters of the structure of the bladder/rectum outside the PTV (NOS) were also obtained. These dosimetric parameters of NOS can be used as plan optimization parameters to participate in planning optimization. So these dosimetric parameters of NOS were also called plan optimization parameters in this paper. Volume of PTV (cm^3^), volume (cm^3^), OV (cm^3^), and OP (%) of bladder/rectum were collected as geometry parameters.

The article "Dose Prediction Models Based on Geometric and Plan Optimization Parameter for Adjuvant Radiotherapy Planning Design in Cervical Cancer Radiotherapy" was retracted in 2023. Reasons: unreliable results or conclusions; concerns about the data; concerns about the peer review; concerns about the citations.

### 2.4. Development and Verification of the Dose Prediction Models

Thirty VMAT plans of the patients were randomly selected for modeling. Correlation of the geometry parameters, corresponding plan optimization parameters of NOS (*V*_30_, *V*_35_, *V*_40_, and *D*_2cc_), and dosimetric parameters (*V*_30_, *V*_35_, *V*_40_, and *D*_2cc_) of bladder/rectum were established, and scatterplots and univariate and multiple linear regression models were employed to explore the association among them.

Ten VMAT plans of patients were randomly selected for verifying the accuracy of the models. Before unknowing the predicted results of using the model, the radiotherapy plans were made by the same physicist until the optimal was considered the best and then the optimization was stopped. The geometry parameters, dosimetric optimization parameters, and dosimetric parameters of bladder/rectum in the radiotherapy planning were extracted using the above methodology from the planning system. These parameters were substituted into the model to calculate the predicted values (*V*_30_, *V*_35_, *V*_40_, and *D*_2cc_) of bladder/rectum. The deviation between the predicted value and the actual planned value was calculated by the following formula: *d* = (D_pre_−*D*_actual_)/*D*_actual_, *D*_pre,_ and *D*_actual_ represent the predicted and actual values, respectively.

### 2.5. Statistical Analysis

Statistical analysis was done using the SPSS 26.0 (IBM, Armonk, NY, USA). Geometry parameters and dosimetric parameters of bladder/rectum and their NOS (i.e., dosimetric optimization parameters) were summarized. Baseline characteristics were presented using the standard descriptive statistics: mean ± standard deviation for the continuous variables with normal distribution. Depending on the data type, initially, the univariate linear regression was used to screen out statistically different influencing factors, and then multiple linear regression was used by the primary influencing factors, excluding collinearity to build the dosimetric prediction models. *P* < 0.05 was considered statistically significant.

## 3. Result

### 3.1. Evaluation of Planning Target Volume Coverage

Table 1 shows the evaluation of the PTV dose coverage of models. Dose *D*_95_ for PTV ranged from 50.3 Gy to 50.6 Gy that was 99.8%–100.3% of the prescribed dose (50.4 Gy), on an average of 50.4 Gy. Dose *D*_2_ for PTV ranged from 53.1 Gy to 54.1 Gy that was 105.3%–107.3% of the prescribed dose (50.4 Gy),, on an average of 53.7 Gy, which was <110% of the prescription dose and limited in the target. Dose *D*_98_ for PTV ranged from 49.4 Gy to 49.9 Gy that was 98%–99% of the prescribed dose (50.4 Gy), which was >95% of the prescription dose. CI varied ranged from 0.82 to 0.93, on average of 0.86. CI above 0.7 was acceptable and consistent with a previous report [27]. HI varied ranged from 0.06 to 0.09, on average of 0.08. PTV volume of each patient was measured using Eclipse TPS.

The article "Dose Prediction Models Based on Geometric and Plan Optimization Parameter for Adjuvant Radiotherapy Planning Design in Cervical Cancer Radiotherapy" was retracted in 2023. Reasons: unreliable results or conclusions; concerns about the data; concerns about the peer review; concerns about the citations.

### 3.2. Dosimetric Sparing of Bladder and Rectum

The dose of bladder/rectum and their NOS is shown in Table 2. *V*_30_ doses of 57.5% in the range of 40.3%–72.9% and 54.1% in the range of 35.2%–70.6% were observed for bladder and rectum, respectively. *V*_35_ doses of 45.9% in the range of 31.8%–60.3% and 41.8% in the range of 24.9%–56.0% were observed for bladder and rectum, respectively. *V*_40_ dose ranged from 25.1% to 52.3%, with an average of 35.7% for the bladder, and 17.8% to 44.8%, with an average of 31.3% for the rectum, respectively.

Dose D_2cc_ ranged from 52.9 Gy to 53.9 Gy that was 104.9%–106.9% of the prescribed dose (50.4 Gy), with an average of 53.4 Gy for the bladder, and 49.9 Gy to 52.8 Gy that was 98.2%–104.8% of the prescribed dose (50.4 Gy), with an average of 51.6 Gy for the rectum. Some plans failed to meet the dose limits of *V*_40_ < 40% in case of the rectum and bladder, because of the large overlap volume of the PTV. In such cases, a compromise was considered between the deficit target and OAR protection.

### 3.3. Dosimetric Prediction Model

The main focus of the present study was the examination of the relationship between the bladder/rectum dosimetric parameters (*V*_30_, *V*_35_, *V*_40_, and *D*_2cc_), the geometry parameters, and the corresponding dosimetric optimization parameters of the nonoverlap bladder/rectum structure. Considering all underlying factors, it was found that the relationship could be described using linear regression formulas. For both bladder and rectum, the univariate linear regression formula was found for D_2cc_: the formulas of bladder and rectum were *D*_2cc_ = 3.66 OP _bladder_ (%) + 5275.19 (cGy) (*R*^2^ = 0.447, *P* < 0.001) and *D*_2cc_ = 22.02 OV _rectum_ (cm^3^) + 5028.97 (cGy) (*R*^2^ = 0.543 *P* < 0.001), respectively (Figure 1). The multiple linear regression was found for *V*_30_, *V*_35_, and *V*_40_ as *Vn* = *A* × OP (%) + *B* × *V*_n-NOS_ + *C*, where *Vn* was the percent volume covered by a dose of at least *n* Gy for bladder/rectum and *V*_n-NOS_ was the percent volume covered by the corresponding dose of at least *n* Gy for the nonoverlap bladder/rectum structure. The values of the multiple linear regression model for the prediction of dose-volume parameters are listed in Table 3. The models of V_40_ for bladder and rectum are shown in Figures 2 and 3. The univariate and multivariate linear regression significance scores of the bladder and rectum are shown in Tables 4 and 5.

The article "Dose Prediction Models Based on Geometric and Plan Optimization Parameter for Adjuvant Radiotherapy Planning Design in Cervical Cancer Radiotherapy" was retracted in 2023. Reasons: unreliable results or conclusions; concerns about the data; concerns about the peer review; concerns about the citations.

The percent volume overlapped with the PTV of bladder/rectum was related to the middose of OAR. The dose-volume parameter *V*_*n*_ of nonoverlapped bladder/rectum structure was related to the corresponding dose of the OAR for guiding the plan design.

### 3.4. Verification of Accuracy of the Model

Ten VMAT plans designed by the same physicist were randomly selected without knowing the laws of these models. Subsequently, the corresponding parameters were imported from these plans into the model to calculate the corresponding dosimetric parameters of bladder/rectum. The actual and calculated dosimetric parameters of bladder/rectum were compared to verify the accuracy of these models. The deviation between the predicted value and the actual planned value was calculated by the following formula: *d* = (*D*_pre_−*D*_actual_)/*D*_actual_, where, *D*_pre_ and *D*_actual_ represent predicted and actual values, respectively. The deviations of these models are listed in Table 6. The average deviations of these dosimetric models ranged from 0.05% to 0.15% in case of the bladder and −0.31% to −0.04% in case of the rectum. The results indicated that the absolute value of these deviations was less than 0.5% and offered a high degree of accuracy. For bladder, the predicted dose was higher than the actual dose, while for rectum, the actual dose was higher than the predicted dose.

## 4. Discussion

Radiation therapy has traditionally been combined with consecutive external beam radiotherapy (EBRT) and intracavitary brachytherapy (ICBT) in the treatment of cervical cancer. ICBT is usually started after EBRT since the OAR near the target is not completely free from the dose during treatment planning [28]. In particular, the dose distribution in the brachytherapy is closely related to the doctor's operation and the patient's preparation state, so it is difficult to ensure the stability of the therapeutic dose each time. The lower the dose of EBRT to the OAR, the greater the dose sparing of the OARs in brachytherapy and the lower the overall dose of the OARs, with fewer potential side effects.

With the development in radiotherapy technology, the inverse planning such as intensity-modulated radiation therapy (IMRT) and volumetric-modulated arc therapy (VMAT) is gradually replacing the traditional relatively simple techniques such as 3D conformal radiation therapy involving complex dose distributions (e.g., convex and concave shapes) [29]. Due to the complexity of the shape and configuration of the tumor and lymph nodes in the target region and close proximity of OAR, IMRT or VMAT has been widely used in treatment planning [30]. VMAT is a new form of IMRT with continuous changeable dose rate, gantry speed, and dynamic multileaf collimator movement [31]. The major advantages of VMAT over IMRT involve the decreased MU and treatment delivery time [32, 33]. Inverse planning allows the planner to set the desired dose objectives, which are used by the optimization algorithm to iteratively search for the optimal machine parameters that meet the desired dose objectives. While inverse planning allows the planners to avoid the need to manually segment each field, the ideal set of the initial dose objectives is subjective and not known a priori. This requires much time and effort to explore, which leads to suboptimal treatment plans and treatment plan quality variations within and across the institutions due to interplanner subjectivity and bias. Planning strategies that reduce planner bias would directly improve the quality and consistency of treatment plans [20, 22, 34, 35]. As a result, a stable and easy-to-control plan design method is necessary.

The article "Dose Prediction Models Based on Geometric and Plan Optimization Parameter for Adjuvant Radiotherapy Planning Design in Cervical Cancer Radiotherapy" was retracted in 2023. Reasons: unreliable results or conclusions; concerns about the data; concerns about the peer review; concerns about the citations.

Some reports have studied the effect of the geometric factors of the patient anatomy such as the OAR size, target volume, and overlap volume on the radiotherapy dose [19, 20, 36–38]. The overlap volume of OAR and target is considered as a key factor primarily affecting the OAR dose. Traditional plan designs mostly limit the dose and volume of the entire OAR structure. However, it is not easy to plan a designing parameter with uniformity and stability in different subjects with different OAR volume, executed by different planners. Our approach involved a simplified method of predicting the noncompliance to OAR constraints by combining the patient anatomical parameters and plan design parameters, and the results can be used to guide the plan designing directly.

For a high-quality plan, the dose line can be seen to drop uniformly outside the target area by the naked eye. It is not easy to operate and ensure that the target area meets the prescribed dose requirement in the plan design if the dose restriction is imposed on the whole OAR. Therefore, there is a need to maximize the protection of the OAR, while not losing the prescribed dose in the target area. Dose restriction is imposed on the nonoverlapping target area of the OARs, wherein a relationship exists between it and the dose. It is also easier to adjust instead of adjusting the entire OAR. There are currently no similar literature reports on the relationship between the nonoverlapping areas and the patient anatomy and dose.

The article "Dose Prediction Models Based on Geometric and Plan Optimization Parameter for Adjuvant Radiotherapy Planning Design in Cervical Cancer Radiotherapy" was retracted in 2023. Reasons: unreliable results or conclusions; concerns about the data; concerns about the peer review; concerns about the citations.

For the geometric parameters, a significant correlation was found between the overlap volume of bladder/rectum and dose, which was in good agreement with the findings of Caine et al. in prostate cancer [36]. In our study, the dose analyzed was related to the percentage overlap volume (OP) and the corresponding dose-volume optimization parameters of nonoverlap volume (NOS) except D_2cc_. Generally, D_2cc_ means dose to the hottest dose to 2 cm^3^ of tissue. It is used in the assessment of the bladder and rectal toxicity, and growing evidence supports that D2cc is one of the most reliable indexes that predicts late morbidities in the rectum or bladder [39–41]. Since the dose to the hottest dose to 2 cm^3^ of bladder/rectum lies only in the overlap volume, there was no significant correlation between the nonoverlap volume (NOS) and *D*2cc. But NOS can be exposed with a dose of 30 Gy, 35 Gy, and 40 Gy, so the dose-volume optimization parameters Vn of bladder/rectum are related to both the overlap volume and NOS.

Earlier studies [18, 19] found the exact relationship between the volume-dosimetric parameters of OAR and patient anatomy-related factors. Honglai Zhang [19] found the unary linear relationship between the parotid (*R*^2^ = 0.95, *P* < 0.0001)/submandibular glands (*R*^2^ = 0.98, *P* < 0.0001) and the mean dose and percent volume overlapped with PTV_58_ in head-and-neck cancer. Also, it was found that the mean dose for the parotid <26 Gy could be achieved with <20% volumetric overlap with PTV_58_ and for submandibular glands (SMGs), an average *D*_mean_ of 27.6 Gy was achieved in patients having <10% overlap with PTV and 36.1 Gy when <20% overlap according to the statistical description. It was found that the dose relationship in our study was related to multiple factors, which means that the dose is influenced by the confluence of different factors, so we only got the ranges and equations instead of the exact cutoff value of these factors. The percentage overlapped volume ranges of the bladder and rectum were 9.11∼29.70% and 5.56∼20.66%, respectively. The *V*_30_, *V*_35_, and *V*_40_ ranges of NOS were 31.3∼65.5%, 21.5∼48%, and 14.6∼30.7%, respectively, for the bladder and 29.2∼65.1%, 19.8∼47.5%, and 12.3∼31.4%, respectively, for the rectum. *R*^2^ of Vn dose prediction models improved to 0.99, when the dose-volume optimization parameters of NOS were added. In the patients, the overlap volume is stable, but the dose-volume optimization parameters of NOS can be adjusted, which can be used to directly guide the plan design compared with other single factor models. As a result, the plan design is more convenient and maneuverable.

The deviation of these models was less than 0.5%, which can prove that the high accuracy of these models and the consistency of the plans are better. However, we found out the predictive value of bladder was higher than the actual value in the mode and the opposite case in the rectum. The bladder and rectum are commonly affected organs and they are the common site of injury following radiotherapy of the pelvic due to its relatively fixed central position in the pelvis. We believe that the bladder and rectum can affect each other as they are anterior and posterior to the uterus. There is a possibility of the occurrence of interactions between the OAR exposed to the same dose. Simultaneously depressing the bladder and rectum dose may cause high doses in the target to affect the uniformity of the target dose. In order to balance the dose among the target and each OAR, some OAR sufficient to meet the dose limit can be relaxed, making room to limit the high dose of other OARs. The next step of this study will be to investigate the dose interaction of target and different OARs.

The article "Dose Prediction Models Based on Geometric and Plan Optimization Parameter for Adjuvant Radiotherapy Planning Design in Cervical Cancer Radiotherapy" was retracted in 2023. Reasons: unreliable results or conclusions; concerns about the data; concerns about the peer review; concerns about the citations.

Although automated plans are growing rapidly, there is a need to apply this knowledge to a simple clinician-oriented metric to aid high-quality plan designing, because a large number of high-quality plans are needed for building a database for developing high-quality automated planning, which is more complicated. It is necessary to input the structural parameters, dosimetric parameters, position parameters, and other pieces of information of the radiotherapy plan. However, the information to be extracted by the automatic learning technology is still unknown and needs exploration.

The new plan can be designed according to the plans in the database; these patients may have similar information about the organ structures, dosage prescription, structure location, and so on. Such knowledge-based planning (KBP) techniques [20, 42, 43] utilize the anatomical and dosimetric information from previously treated patients to guide the planning for a new patient. KBP methods query a new patient against a retrospective patient database for a subset of patients with similar anatomy and use the dose data from the queried database patients to inform the planning of the new patient [20]. These methods are more complex and costly and there is a need to support the plan assessment with external quantitative tools to better understand the available potential. There are certain defects in this study; for instance, the study did not consider the fact that the bladder or rectum does not overlap the target area at all and the geometric parameters considered only contain the overlap (bladder/rectum versus PTV) volume, without considering the OAR shape, orientation, or geometric irregularities. These situations and the effects among different OAR need more research. The radiotherapy plans used for model establishment in the study were designed by the only physicist with senior professional title in our institution, who has nearly 10 years of radiotherapy plan design experience and is considered to be the physicist with the highest level of plan design in our institution. The robustness of the model requires further internal and external validation in the next step. In this study, we were surprised to find this law and proposed this model. It can be more direct and convenient to guide plan design. In the next step, we hoped that this method can be helpful to solve the current planning level differences between different physicists and different institutions to improve plan quality quickly. The next stage of the research is to comprehensively improve and verify the stability of the model from both internal and external perspectives and further improve the accuracy and stability of the model by combining the plan design experience of different people and institutions.

The article "Dose Prediction Models Based on Geometric and Plan Optimization Parameter for Adjuvant Radiotherapy Planning Design in Cervical Cancer Radiotherapy" was retracted in 2023. Reasons: unreliable results or conclusions; concerns about the data; concerns about the peer review; concerns about the citations.

There are other effective factors reported such as whether there is lymph node metastasis [36, 38], different prescription doses [7, 18], and the volume of the organs in the field [20]. These can be added to the model in future research to optimize the models and expand the scope of use of the models. The linear relationship we found between the dose of OAR, OAR volume overlapped with PTV, and nonoverlap volume structure dose can be used as a basis to establish automated planning. The quality and consistency of the VMAT plan in cervical cancer are more important for automated planning. Knowledge-based planning has become more popular in radiation therapy in recent years. To apply machine learning techniques, the creation of automated planning model becomes essential [44, 45]. The plan quality is dependent on the applied database quality, in which overlap volume is considered to be a major factor [20, 46–49]. The dosimetry parameters of nonoverlap volume structure make it easier to establish a high-quality and homogeneous plan database. The results of the current work could potentially be applied for developing automated planning and resolving the problem of inconsistent planning experience among different planners and different institutions. Further steps of this study include the application of the models among different plan designers and agencies to verify their effectiveness, homogeneity of plan quality, developing models for different dosage prescriptions, and establishing automatic plan models.

## 5. Conclusion

This study shows that there is a linear relationship between the dose of the bladder/rectum, their percent overlap volume with the PTV, and corresponding dosimetric optimization parameters of their nonoverlapping structure. Compared with other researches, multivariate mathematical models in our study consider the new influencing factors (dosimetric optimization parameters for nonoverlapping structure). The linear relationship can predict the dose similar to other studies, but the difference is that the dosimetric optimization parameters for nonoverlapping structure included in our models also can be used to guide the plan design directly in planning optimization process. It makes planning optimization more flexible and convenient and the model more clinically practical. This can assure a sufficient target dose, which can facilitate the speed of the optimization process and unify and stabilize the plan quality.

The article "Dose Prediction Models Based on Geometric and Plan Optimization Parameter for Adjuvant Radiotherapy Planning Design in Cervical Cancer Radiotherapy" was retracted in 2023. Reasons: unreliable results or conclusions; concerns about the data; concerns about the peer review; concerns about the citations.

## Figures and Tables

**Figure 1:** (a, b) Univariate linear relationship of bladder (a)/rectum (b) *D*_2cc_ and percent volume/volume overlapped with PTV. ^*∗*^Increase of *D*_2cc_ was correlated with the percent overlap volume/volume increased. The linear relationship was statistically significant (*P* < 0.001).

**Figure 2:** Multiple linear regression model for dose *V*_40_ prediction of the bladder. ^*∗*^Multiple linear regression model for the dose *V*_40_, the percent volume overlapped with PTV (OP_bladder_), and *V*_40_ for the nonoverlapped structure of bladder (*V*_40-NOSbladder_) are shown. Level of statistical significance was *P* < 0.001.

**Figure 3:** Multiple linear regression model for dose *V*_40_ prediction of the rectum. ^*∗*^Multiple linear regression model for the dose *V*_40_, percent volume overlapped with PTV (OP_rectum_), and *V*_40_ for the nonoverlapped structure of rectum (*V*_40-NOSrectum_) are shown. Level of statistical significance was *P* < 0.001.

**Table 1:** Planning target volume dose coverage.

	*D*_95_, cGy	*D*_2_, cGy	*D*_98_, cGy	CI	HI	Volume, cm^3^
Average	5040.54	5368.94	4966.95	0.86	0.08	868.14
SD	7.22	24.47	11.74	0.03	0.01	112.63

**Table 2:** Dosimetric parameters and volume of bladder and rectum.

	Bladder	Rectum	NOS bladder	NOS rectum
Volume, cm^3^	260.15 ± 74.26	54.38 ± 18.68	216.78 ± 69.73	47.49 ± 17.01
V_30_, %	57.54 ± 7.23	54.05 ± 9.15	48.71 ± 7.29	47.29 ± 9.31
V_35_, %	45.86 ± 7.16	41.78 ± 7.69	34.64 ± 5.77	33.16 ± 6.86
V_40_, %	35.74 ± 6.82	31.33 ± 6.27	22.40 ± 3.90	21.14 ± 4.62
D_2cc_, Gy	5336.03 ± 30.86	5162.26 ± 71.66	4968.22 ± 74.68	4704.50 ± 105.95
Volume percent	1.00	1.00	0.83 ± 0.06	0.87 ± 0.04

NOS bladder represents the structure of the bladder out of PTV. NOS rectum represents the structure of the rectum out of PTV.

The article "Dose Prediction Models Based on Geometric and Plan Optimization Parameter for Adjuvant Radiotherapy Planning Design in Cervical Cancer Radiotherapy" was retracted in 2023. Reasons: unreliable results or conclusions; concerns about the data; concerns about the peer review; concerns about the citations.

**Table 3:** Values of the multiple linear regression model for prediction of dose-volume parameter.

	*V*_*n*_	A	B	C	R^2^
Bladder	*V*_30_	0.511	0.843	7.966	0.997
	*V*_35_	0.646	0.853	5.588	0.997
	*V*_40_	0.771	0.840	4.108	0.997

Rectum	*V*_30_	0.557	0.886	5.754	0.997
	*V*_35_	0.669	0.916	3.746	0.995
	*V*_40_	0.783	0.953	2.223	0.993

*V*_*n*_ = *A* × OP (%) + *B* × *V*_*n*-NOS_ + *C. V*_n_: the percent volume covered by a dose of at least *n* Gy for bladder/rectum. *V*_*n*-NOS_: the percent volume covered by the corresponding dose of at least *n* Gy for the nonoverlap bladder/rectum structure. OP: overlapped volume as a percentage of bladder/rectum volumes A, B, and C are regression constants.

**Table 4:** Univariate and multivariate linear regression significance scores for prediction of the bladder dose.

Variables	Outcome	*P* value	*R* ^2^	*P* value	*R* ^2^
	variable	(univariate)	(univariate)	(multivariate)	(multivariate)
PTV volume	*V*_30_	0.039	0.113	0.869	0.997
	*V*_35_	0.038	0.114	0.976	0.997
	*V*_40_	0.036	0.117	0.936	0.997
	D2cc	0.006	0.215	0.167	0.467

Bladder volume	*V*_30_	0.088	0.068	N	N
	*V*_35_	0.032	0.123	0.351	0.997
	*V*_40_	0.028	0.13	0.403	0.997
	D2cc	0.631	0.027	N	N

OV^*∗*^ of bladder	*V*_30_	0.099	0.062	N	N
	*V*_35_	0.015	0.165	N	N
	*V*_40_	0.001	0.288	N	N
	D2cc	0.002	0.26	N	N

OP^*∗*^ of bladder	*V*_30_	0.002	0.266	<0.001	0.997
	*V*_35_	<0.001	0.57	<0.001	0.997
	*V*_40_	<0.001	0.83	<0.001	0.997
	D2cc	<0.001	0.447	<0.001	0.467

*V*_30_ of NOS bladder^*∗*^	*V*_30_	<0.001	0.83	<0.001	0.997
*V*_35_ of NOS bladder^*∗*^	*V*_35_	<0.001	0.754	<0.001	0.997
*V*_40_ of NOS bladder^*∗*^	*V*_40_	<0.001	0.69	<0.001	0.997
D2cc of NOS bladder^*∗*^	D2cc	0.861	0.035	N	N

^∗^OV: the volume of the overlap of the OAR with the PTV; OP: the percentage volume of the overlap of the OAR; NOS bladder: the structure of the bladder outside the PTV; N indicated that this parameter did not participate in the multivariate linear regression analysis.

**Table 5:** Univariate and multivariate linear regression significance scores for prediction of the rectum dose.

Variables	Outcome	*P* value	*R* ^2^	*P* value	*R* ^2^
	variable	(univariate)	(univariate)	(multivariate)	(multivariate)
PTV volume	*V*_30_	0.057	0.092	N	N
	*V*_35_	0.151	0.039	N	N
	*V*_40_	0.378	0.028	N	N
	D2cc	0.772	0.033	N	N

Rectal volume	*V*_30_	0.235	0.016	N	N
	*V*_35_	0.197	0.025	N	N
	*V*_40_	0.212	0.021	N	N
	D2cc	0.036	0.117	N	N

OV*∗* of rectum	*V*_30_	0.235	0.016	N	N
	*V*_35_	0.068	0.082	N	N
	*V*_40_	0.017	0.156	0.266	0.993
	D2cc	<0.001	0.543	<0.001	0.543

OP*∗* of rectum	*V*_30_	0.002	0.26	<0.001	0.997
	*V*_35_	<0.001	0.454	<0.001	0.995
	*V*_40_	<0.001	0.612	<0.001	0.993
	D2cc	0.002	0.272	N	N

V30 of NOS rectum*∗*	*V*_30_	<0.001	0.955	<0.001	0.997
V35 of NOS rectum*∗*	*V*_35_	<0.001	0.919	<0.001	0.995
V40 of NOS rectum*∗*	*V*_40_	<0.001	0.843	<0.001	0.993
D2cc of NOS rectum*∗*	D2cc	0.008	0.196	0.811	0.527

*∗* ^∗^OV: the volume of the overlap of the OAR with the PTV; OP: the percentage volume of the overlap of the OAR; NOS rectum: the structure of the rectum outside the PTV; N indicated that this parameter did not participate in the multivariate linear regression analysis.

The article "Dose Prediction Models Based on Geometric and Plan Optimization Parameter for Adjuvant Radiotherapy Planning Design in Cervical Cancer Radiotherapy" was retracted in 2023. Reasons: unreliable results or conclusions; concerns about the data; concerns about the peer review; concerns about the citations.

**Table 6:** Statistical analysis of % accuracy deviation of the models.

		*V*_30_, %	*V*_35_, %	*V*_40_, %	D2cc, cGy
Bladder	D_pre_	56.66 ± 8.24	43.74 ± 5.86	33.32 ± 4.54	5332.45 ± 8.92
	D_actual_	56.59 ± 8.30	43.73 ± 5.89	33.30 ± 4.65	5329.05 ± 30.18
	Deviation (%)	0.15 ± 0.57	0.05 ± 0.7	0.13 ± 0.86	0.07 ± 0.49

Rectum	D_pre_	57.06 ± 11.84	41.73 ± 8.27	30.67 ± 7.40	5123.21 ± 28.16
	D_actual_	57.06 ± 11.61	41.82 ± 8.28	30.80 ± 7.60	5132.47 ± 81.44
	Deviation (%)	− 0.04 ± 1.3	− 0.19 ± 1.56	− 0.31 ± 2.26	− 0.16 ± 1.12

## Data Availability

The data used to support the study are available from the corresponding author upon request.
